The article "A Gray Correlation Algorithm for Analysis of Influencing Factors of Film and Television Copyright Export" was published in 2022. Journal: Comput Intell Neurosci.

# A Gray Correlation Algorithm for Analysis of Influencing Factors of Film and Television Copyright Export

**DOI:** 10.1155/2022/3510552

**Published:** 2022-03-16

**Authors:** Bingchao Ren, Ting Jin

**Affiliations:** ^1^School of Intellectual Property, Nanjing University of Science & Technology, Nanjing 210094, China; ^2^School of Literature, Journalism & Communication, Henan University of Economics and Law, Zhengzhou 450046, China; ^3^School of Journalism and Communications, Henan University of Technology, Zhengzhou 450001, China

## Abstract

In this paper, an intelligent model is constructed to facilitate real-time dynamic analysis of the factors affecting the export of film and television copyrights and to track the process of spatiotemporal context. The algorithm analyzes the factors affecting the export of film and television copyrights according to actual needs. Through the comparative analysis of experimental models, the influence and optimization of gamma correction and Laplace distribution weighting on spatial context information and confidence map update are verified. In addition, this paper uses the gray relational algorithm to construct an analysis system of factors affecting the export of film and television copyright. The research shows that the analysis model of the influencing factors of film and television copyright export based on the gray relational algorithm can play a very good role in the analysis of these factors.

## 1. Introduction

In the new normal economic environment, there is no doubt that China's export structure also needs supply-side reforms. In terms of film and television cultural works, our country has been in a state of deficit in international trade for a long time. With the development of economy, people began to pursue spiritual and cultural life after satisfying their material life. With the transformation of society and changes in consumption concepts and lifestyles, as well as the promotion of technological factors such as Internet technology and new media technology, film and television cultural works appear more and more frequently in people's lives, and people's expenditure on film and television cultural works is also increasing.

On the one hand, as a kind of copyright, film and television copyright has the characteristics of copyright, which can be summarized into three types: “exclusiveness,” “territoriality,” and “timeliness.” “Exclusivity” means that copyright is as exclusive as ownership. Copyright is exclusively owned by the right holder, and this right of the right holder is strictly protected by law. Moreover, in addition to the exceptions provided by the law, the use of the work by others must obtain the permission of the right holder. “Territoriality” means that the effectiveness of copyright is restricted by space and only extends to the territory of the country, which is strictly territorial. Unless international conventions or bilateral treaties are signed between countries, intellectual property rights do not have extraterritorial effects, and anyone outside of the country can freely use the copyright. However, due to the accelerating process of today's world integration and the increasingly frequent exchanges between countries, transnational copyrights and transnational jurisdictions of copyrights and worldwide intellectual property protection organizations have emerged. Therefore, the characteristic of “territoriality” is gradually diminishing [1]. “Timeliness” means that the protection of copyright is limited by time. If the copyright exceeds the copyright protection period stipulated by law, it will no longer be protected. Generally speaking, the authorship right, the right to modify and, the right to protect the integrity of the work in the personal rights of copyright are not restricted by time and will not disappear due to the death of a person. The right of publication in property rights and personal rights is restricted by the term of copyright protection [2]. On the other hand, film and television copyright also has its own characteristics. Film and television works are a collection of independent works such as music, songs, scripts, audio, and video. It is based on these independent works as a whole formed through the processing of modern technology and takes the whole as the object of copyright protection. At the same time, these independent works are separately protected by the law, and the protection of the copyright of these works does not prevent the film and television works as a whole from being protected by the law. Therefore, there is a unique problem of multiple copyrights in the protection of film and television copyrights [3].

In order to facilitate the analysis of the factors affecting the export of film and television copyrights, this paper constructs an intelligent model for real-time analysis of the factors affecting the export of film and television copyrights, which provides a theoretical reference for subsequent related research.

## 2. Related Work

In international trade, cultural trade is extremely special. It is based on cultural industries and involves trade in goods, trade in services, and intellectual property rights. The International Monetary Fund (IMF) describes international cultural trade as exchanges between countries and between residents and nonresidents, and personal, cultural, and entertainment service transactions are all within the category of cultural trade. It is subdivided into the following two categories: one is audiovisual and related services, and the other is other cultural and entertainment services [4].

The rise of cultural trade has attracted the attention and research of many economists, hoping to find a theoretical basis that can explain cultural trade [5]. Literature [6] believes that traditional trade theory can explain the rise of cultural trade. For example, the United Kingdom has a comparative advantage in Shakespeare's plays, and the United States has a comparative advantage in movies, so that the two countries can exchange works with each other. The United Kingdom concentrates on producing and exporting dramas and importing relatively disadvantaged movies, while the United States concentrates on producing and exporting movies and importing dramas. In this way, both countries can gain benefits in international trade. Literature [7] believes that traditional trade theories such as comparative advantage theory and factor endowment theory are more suitable for imitable cultural products. For example, the labor force in developing countries is relatively surplus and has a comparative advantage in the production of imitable cultural products, so that the export of labor-intensive cultural products can be profitable. However, traditional trade theories have no explanatory power for the trade of cultural products that cannot be imitated.

Literature [8] believes that there are external economies of scale in the cultural industry and the agglomeration of producers in the geographic location forms a large-scale operation. Several film and television companies in Hollywood, the United States, have concentrated on all the links of film production, showing a highly vertical integration situation and forming an efficient external scale economy effect. This vertical integration can achieve large-scale operations; reduce unnecessary market circulation links, thereby reducing production costs; and help companies integrate their own advantages, realize resource sharing, and achieve good economic benefits. Literature [9] believes that there are also internal economies of scale in the cultural industry. Take the production of movies as an example. Copying ready-made templates can greatly reduce the production costs of movies. Large-scale film and television groups integrate small-scale scattered resources to reduce production costs in production, so as to obtain cost advantages in competition, thereby forcing small companies to withdraw from the market and gaining market share.

Literature [10] puts forward the so-called first actor advantage theory while considering the effect of economies of scale on international cultural trade. Literature [11] argues that the reason why the United States can occupy an absolute share of the global TV market and continuously export cultural products to the outside world is that it has economies of scale and first actor advantages. Large-scale production has given American TV production companies a stronger cost advantage, with the ability to share fixed costs; product upgrades; and relatively sufficient funds required for advertising, making it a greater advantage in the competition of similar cultural products. The first actor advantage considers certain technical conditions, and through actions such as first improving management, increasing labor productivity, improving marketing channels, and being familiar with the market conditions of the exporting country, American cultural production companies can obtain a “leading” advantage in the production of cultural products [12].

Literature [13] applies demand preference theory to cultural trade. Literature [14] believes that the consumption of cultural products can be understood as the satisfaction that people get from current consumption and the accumulation of future knowledge and experience. Therefore, the past consumption structure of cultural products largely determines the future consumption structure.

Literature [15] believes that the theory of comparative advantage can be used to analyze cultural trade. Literature [16] believes that factor endowments, production technology, production methods, and innovation capabilities can cultivate the comparative advantages of the cultural industry. With these comparative advantages, cultural trade can be carried out. Literature [17] used the theory of comparative advantage to explain cultural trade, specifically pointing out that the main advantages of cultural industry participating in international trade are the resource endowment on the supply side, the advantages of knowledge and technology, and the scale of demand.

Literature [18] agrees that the theory of economies of scale is applicable to cultural trade. Take American movies as an example; the formation of Hollywood has reduced the production and production costs of American movies to a large extent. This specialized assembly line and industrial chain have enabled American movies to dominate the world and win high profits. Literature [19] points out that cultural trade is intraindustry trade and uses demand preference theory to analyze it. The vast majority of international trade in cultural products is carried out between a few countries and is highly concentrated in a few countries, which is a typical intraindustry trade. The theory of preference similarity can explain the phenomenon that the import and export of international cultural trade are highly concentrated between European and American countries with a common cultural background and between the United States and Canada in North America [20].

## 3. Factor Analysis Model Based on Gray Relational Algorithm

This paper mainly analyzes the influencing factors of film and television copyright export through gray relational algorithm and improves it based on the kernel *K*-means algorithm. By taking the nonlinear constraint of the kernel *K*-means algorithm as a penalty term, that is, taking the last term of the constraint in the formula as an independent penalty term, it is combined with the kernel *K*-means clustering algorithm. In order to extract more effective information in the process of clustering, orthogonality constraints and nonnegativity constraints are added to the proposed model at the same time, and the improved penalized K-means clustering model (PKKM) is obtained in this paper. The objective function is as follows:

(1) $$\begin{array}{c} \underset{H}{\max}Tr\left[H^{T}KH\right]-\alpha {\left\|1_{n}^{T}-1_{n}^{T}HH^{T}\right\|}_{F}^{2},\\ s.t.\;H\geq 0,H^{T}H=I. \end{array}$$

Among them, *K* represents the kernel matrix, and *α* is a hyperparameter.

When H satisfies the orthogonality constraint, based on the properties of the Frobenius function and the trace function, the penalty term in (1) can be written as follows:

(2) $$\begin{array}{c} {\left\|1_{n}^{T}-1_{n}^{T}HH^{T}\right\|}_{F}^{2}=Tr\left[1_{n}1_{n}^{T}\right]-Tr\left[H^{T}1_{n}1_{n}^{T}H\right]. \end{array}$$

Therefore, (1) can be written in the following form:

(3) $$\begin{array}{c} Tr\left[H^{T}KH\right]-\alpha {\left\|1_{n}^{T}-1_{n}^{T}HH^{T}\right\|}_{F}^{2},\\ =Tr\left[H^{T}KH\right]+\alpha Tr{\left\|H^{T}1_{n}1_{n}^{T}H\right\|}_{F}^{2}-\alpha Tr\left[1_{n}1_{n}^{T}\right],\\ =Tr\left[H^{T}\left(K+\alpha E\right)H\right]-\alpha n. \end{array}$$

Among them, *E*=1_*n*_1_*n*_^*T*^ represents an *n* ×*n* matrix, and all elements in the matrix are 1.

Because the proposed PKKM model has orthogonal and nonnegative constraints, in the process of optimizing the above objective function, the nonconvexity of the model itself makes the solution of the model an NP-hard problem. Therefore, this paper proposes a simple but robust numerical algorithm. The algorithm splits the original matrix variable into two variables through the splitting method and satisfies the orthogonality and nonnegativity constraints. The problem of solving the objective function is transformed into a problem of seeking extreme values of two variables. Furthermore, the algorithm uses an alternate iteration method to find solutions that meet the constraints. The split model is a more relaxed model. The objective function of the model is as follows [21]:

(4) $$\begin{array}{c} \underset{x,H}{\max}Tr\left[H^{T}\left(K+\alpha E\right)H\right]-\frac{\mu }{2}{\left\|H-X\right\|}_{F}^{2},\\ s.t\text{. }H\geq 0,H^{T}H=I. \end{array}$$

Among them, the second term in formula (2) can be written as follows:

(5) $$\begin{array}{c} \frac{\mu }{2}{\left\|H-X\right\|}_{F}^{2},\\ =\frac{\mu }{2}\left({\left\|X\right\|}_{F}^{2}-2Tr\left[H^{T}X\right]+{\left\|H\right\|}_{F}^{2}\right),\\ =\frac{\mu }{2}{\left\|X\right\|}_{F}^{2}-Tr\left[H^{T}\left(\mu I\right)X\right]+\frac{\mu k}{2}. \end{array}$$

Therefore, the solution to the subproblem of *H* in the above problem can be described as follows:

(6) $$\begin{array}{c} \underset{H}{\max}\left[H^{T}\left(\mu I\right)X\right]\text{,}\\ \mathrm{s.t.}\;H^{T}H=I\text{.} \end{array}$$

Among them, *K*=*K*+*αE*+*μI*.

The above-mentioned problem is also called the orthogonal Plucker problem, which has a closed-form solution. Below, we solve it by alternating iterative method.

When the variable *X* is fixed, the original problem is transformed into the following: for any matrix *A* ∈ *R*^*n*×*k*^, the objective function of the related optimization problem for *H* ∈ *R*^*n*×*k*^ is as follows:

(7) $$\begin{array}{c} \underset{H}{\max}Tr\left[H^{T}A\right],\\ s.t\text{. }H^{T}H=I. \end{array}$$

Formula (5) has a corresponding closed-form solution:

(8) $$\begin{array}{c} H^{*}=U\left(:,1:k\right)V^{T}. \end{array}$$

Among them, *A*=*U*∑*V*^*T*^ is the singular value decomposition of *A*.

The relevant proof is as follows:

First, *A*=*U*∑*V*^*T*^ is the singular value decomposition of *A*, and the solution of the *H* subproblem is as follows:

(9) $$\begin{array}{c} H^{*}=\underset{H}{\arg\max}Tr\left[H^{T}A\right]\\ =\underset{H}{\arg\max}Tr\left[U\sum V^{T}\right]\\ =\underset{H}{\arg\max}Tr\left[{\left(U^{T}HV\right)}^{T}\sum \right]\\ =U\left(\underset{H}{\arg\max}Tr\left[H^{T}\sum \right]\right)V^{T}\\ =U\left[\begin{array}{c} I_{k}\\ 0 \end{array}\right]V^{T}. \end{array}$$

The solution to the *X* subproblem is as follows: when the orthogonal matrix *H* cannot satisfy the nonnegativity constraint, the update rule for *X* is as follows:

(10) $$\begin{array}{c} X=\max\left(0,H\right). \end{array}$$

Therefore, the entire process above is to update the variables between the Stiefel manifold and the nonnegative quadrant.

In this part, we will discuss the relationship between the proposed PKKM algorithm and some commonly used classic clustering algorithms, such as classic K-means algorithm, orthogonal nonnegative matrix factorization (ONMF) algorithm, spectral clustering, and projection nonnegative matrix factorization (PNMF) algorithm.

This relationship is shown in Figure 1. As can be seen from the figure, compared to the other three clustering algorithms, the model proposed in this paper is the closest relaxation model to the *K*-means model, and its scalability can be changed according to its model. The following part will discuss the relationship between PKKM model and K-means model, ONMF model, spectral clustering, and PNMF model.

When *α*=+*∞*, the PKKM algorithm is equivalent to the *K*-means clustering algorithm.

In the PKKM model, when the parameter *α*=+*∞* of the penalty term in (1) is met, and the constraint condition 1_*n*_^*T*^ − 1_*n*_^*T*^*HH*^*T*^=0 is satisfied at the same time, (1) can be written in the following form:

(11) $$\begin{array}{c} \underset{H}{\max}Tr\left[H^{T}KH\right],\\ s.t\text{. }H\geq 0,H^{T}H=I_{k},1_{n}^{T}-1_{n}^{T}HH^{T}=0. \end{array}$$

Formula (9) is equivalent to the objective function formula of the kernel K mean value.

When the parameter of the penalty term in (1) is *α* = 0, the PKKM model can be written in the following form:

(12) $$\begin{array}{c} \underset{H}{\max}Tr\left[H^{T}KH\right],\\ s.t\text{. }H\geq 0,H^{T}H=I_{k}. \end{array}$$

Equation (12) corresponds to the ONMF model.

Spectral clustering is the orthogonal relaxation of the proposed PKKM model. The objective function of the spectral clustering model is as follows:

(13) $$\begin{array}{c} \underset{X}{\max}Tr\left[X^{T}LX\right],\\ s.t\text{. }X^{T}X=I_{k}. \end{array}$$

In formula (13) of the PKKM model, the kernel matrix *K* + *aE* in the model is replaced by *L*, and then the nonnegativity constraint in the model is removed. Then, the objective function of PKKM is equivalent to the model of spectral clustering.

The PNMF algorithm is a nonnegative relaxation of the proposed PKKM algorithm, and its objective function is as follows:

(14) $$\begin{array}{c} \underset{x\geq 0}{\max}{\left[M-{\text{MXX}}^{T}\right]}_{F}^{2}. \end{array}$$

In formula (1) of the PKKM model, *α* = 0, and the orthogonality constraint is removed; then, the PKKM model and the PNMF model are equivalent.

## 4. Analysis of Influencing Factors of Film and Television Copyright Export Based on Gray Relational Algorithm

The export destinations of Chinese movies are mainly concentrated in two types of countries. One type is Southeast Asian and East Asian countries, which are close to our country's cultural distance and can have a better understanding of Chinese movies. Therefore, in the early stage of our country's film export, works were mainly exported to Southeast Asia, North Korea, and other countries. The other type is European and American countries, which have a developed domestic market and a wealth of domestic works, so there is not much demand for Chinese works. However, due to the relatively developed economies of European and American countries and the demand of local Chinese for domestic films, domestic films can also have some overseas income in Europe and the United States.

The film and television copyright management system creates an end-to-end streaming media content protection platform, while providing all the services needed from the content preparation stage to the delivery stage. The function flow chart of the film and television copyright management system is shown in Figure 2.

The film and television copyright management system uses the HLS protocol for video transmission. The HLS protocol is a streaming media transmission protocol based on HTTP, which can be used to realize video playback on terminal devices. It differs from the common RTP/RTCP and RTSP in that the client-side algorithm obtains complete media content. The content transmitted by HLS mainly includes M3U8 description files and continuous, equal-length TS format media files. Then, it uses the index file of M3U8 to play. The HLS work flow chart is shown in Figure 3.

The copyright tracking system of film and television works will extract and track the feature codes of the film and television works in the library to timely understand the relevant infringement status of the works on the Internet, provide a direction for combating copyright infringement of works, and provide technical support for the copyright protection of film and television works.

After analyzing the needs of the copyright tracking system for text works, it is determined that the system is divided into the following three major modules: infringement information collection, statistical analysis, and auxiliary function modules. Among them, the collection of infringement information is a necessary function, which mainly includes the functions of system importing works, feature code extraction, web crawlers to collect infringement information, and related process scheduling. The statistical analysis module mainly displays some analyzed data, mainly including functions such as hot infringement list, work infringement information query, and infringement information list. The auxiliary function module mainly configures some data of the system operation module, including authorized website management, key monitoring website management, parameter configuration, and domain name information management. The specific system function module structure diagram is shown in Figure 4.

Aiming at solving the problem of information asymmetry between the seller and the authorized party during the transaction of digital works, a trusted counting mechanism is proposed, as shown in Figure 5. Under this mechanism, trusted counters are introduced into the authorized party (authorization system), seller (sales system), and trusted third party (digital work transaction management platform system). Under the combined effect of the three counters, the supervision of digital works transactions is realized. After the sales system receives the order, it extracts the transaction information (including transaction time, seller ID, content provider ID, price, transaction quantity, and digital copyright identification) in the order and then calls the trusted counter of the sales-oriented system for processing. The sales system trusted counter first checks whether the format of the incoming data is legal and generates a transaction request number and a sales random number. Then, it assembles the data into sales permission request data according to the communication protocol in the counter and then signs the sales permission request data to form uploaded data. Finally, it puts the uploaded data into the data buffer pool, and finally the uploaded data is sent to the trusted counter for the management platform through the network. The authorization system obtains authorization-related information (including order information and authorization time) from the outside and calls a trusted counter for the authorization system to process the data. The trusted counter for the authorization system first checks whether the format of the incoming data is legal and generates an authorized random number. Then, the data is assembled into sales license data according to the communication protocol in the counter, and then the sales license data is signed to form upload data. Finally, the uploaded data is put into the data buffer pool and sent to the trusted counter for the management platform through the network. After the trusted counter in the trusted third party receives the uploaded data from the authorized end and the sales end, it first authenticates the data; the data that fails the authentication will be written into the log, and the data that is successfully authenticated will also be matched with the transaction data. Transaction data matching aims mainly to determine whether two uploaded data items belong to the same transaction. If the matching is successful, the uploaded data will be put into the matching database. If the matching fails, the uploaded data will be placed in the unmatched database. In addition, since there are locally generated random numbers in the two types of uploaded data, a certain degree of uniqueness of the data can be guaranteed, and the data signature can ensure the nonrepudiation of the data. Therefore, the mechanism in Figure 5 is credible.

Figure 6 is a schematic diagram of the overall business architecture where the trusted counting system is located. The trusted counter for the sales system, the trusted counter for the authorization system, and the trusted counter for the platform constitute the trusted counting system. The trusted counter for the sales system is used by content sellers. The main function is to complete its own configuration, test the connectivity with the platform counter, complete the processing of transaction information, and upload it to the trusted counter for the platform. The trusted counter for the authorization system is used by integrators and content providers. In addition to completing its own configuration, connectivity testing, and uploading authorization data, it also supports querying the sales records of content sellers. The platform-oriented trusted counter is mainly responsible for the receipt, authentication, and final storage of the data uploaded by the sales and authorized ends (calling the relevant database interface). In addition, it is also responsible for managing the configuration information and usage status of the trusted counter for the sales system and the trusted counter for the authorization system and provides data for the sales record query of the authorized end (calling the relevant data query interface). The trusted transaction management platform conducts statistical supervision of transactions and provides external query services based on the data provided by the trusted counting system.

Figure 7 is a schematic diagram of the digital content publishing business process. First, the publishing unit processes the resources to be released and then releases it to the content provider. After the content provider obtains the resource, according to the nature of the resource and its own situation, it will carry out digital content services through direct sales or consignment by channel dealers. In the case of direct selling, the content provider acts as a content seller at the same time and directly deals with users. There is no issue of credible counting involved here. In the case of consignment sales by channel dealers, content providers have no control over content sellers. At this time, the role of a trusted counting mechanism is needed to help regulators supervise the transactions of data works through three types of counters: trusted counters for sales systems, trusted counters for authorization systems, and trusted counters for platforms. Users (including individual readers and institutions) obtain digital content through purchase and payment, and read or use it through a certain method (designated reading software). Throughout the transaction process, the supervisor monitors the information provided by the trusted counting system to ensure the fairness and credibility of the transaction.

On the basis of the above subsystems, this paper combines the gray correlation algorithm to analyze the factors affecting the export of film and television copyright and constructs the intelligent factor analysis model shown in Figure 8.

After constructing the above model, this paper evaluates the real-time monitoring effect of the film and television copyright export of this system and obtains the results shown in Table 1 and Figure 9.

On the basis of the above analysis, this article evaluates the measured effect of the analysis model of the influence factors of film and television copyright export based on the gray correlation algorithm, and the results are shown in Table 2 and Figure 10.

From the above research, it can be seen that the analysis model of influencing factors of film and television copyright export based on gray correlation algorithm proposed in this paper can play a certain role in the analysis of these factors.

Through the analysis of the above model, we can see that different influencing factors have inconsistent degrees of influence on the import and export of our country's film and television cultural works. The increase in the number of movie screens represents the rapid development of our country's movie market in recent years, which means that the Chinese market's demand for film and television cultural works has increased significantly. Moreover, domestic works can no longer meet the needs of the expanding market and consumers, so it is necessary to continuously import excellent works from abroad. The increase in the enrollment rate of higher education means that there are more people with higher education who have a stronger ability to consume spiritual and cultural products. Therefore, it will also increase the consumer group and consumption of film and television cultural works. In addition, other economic factors such as GDP, technological factors of Internet penetration rate, national policy factors of cultural undertakings, and growth of internal factors such as the number of movies and TV series will cause an increase in the import of film and television cultural works through their respective influence channels. Among the many influencing factors, the GDP growth rate has the strongest correlation with the export of film and television cultural works. The GDP growth rate reflects China's economic growth rate. Although it is a macroeconomic indicator, the overall economic development is an economic environment for a small industry, which will also have a corresponding impact on its export volume.

## 5. Conclusion

Film and television copyright owners will be subject to certain restrictions in the process of exercising film and television copyrights. All countries in the world, including China with its copyright laws, have set certain restrictions on the exercise of copyright. It is mainly reflected in three legal systems: the fair use system, the statutory license system, and the compulsory license system. The fair use system is a basic system of copyright law. It refers to a system where the law allows others to freely use copyrighted works under certain conditions without having to obtain the copyright owner's consent or paying the copyright owner. The factors affecting the export of film and television copyright will continue to change with changes in the general environment, so they need to be studied in light of the actual situation. In order to facilitate the analysis of the export influencing factors of film and television copyright, this paper constructs an intelligent model for real-time analysis of these factors, which provides theoretical reference for subsequent related research. The research results show that the analysis model of film and television copyright export influencing factors proposed in this paper based on the gray correlation algorithm can play a certain role in the analysis of these factors.

## Figures and Tables

**Figure 1:** The relationship between PKKM algorithm and other clustering models.

**Figure 2:** Function flow chart of film and television copyright management system.

**Figure 3:** HLS flow chart.

**Figure 4:** System function module structure diagram.

**Figure 5:** Trusted counting mechanism framework.

**Figure 6:** The overall business architecture where the trusted counting system is located.

**Figure 7:** Digital content publishing business process.

**Figure 8:** Analysis model of influencing factors of film and television copyright export based on gray relational algorithm.

**Figure 9:** Statistical visual chart of the real-time monitoring effect of film and television copyright export.

**Figure 10:** Visual diagram of the actual measurement effect of the analysis model of the factors affecting the export of film and television copyright based on the gray correlation algorithm.

**Table 1:** Real-time monitoring effect of film and television copyright export.

Number	Copyright monitoring
1	93.79
2	94.80
3	92.54
4	92.49
5	86.37
6	94.01
7	89.61
8	84.15
9	93.48
10	94.22
11	85.64
12	93.89
13	86.50
14	85.78
15	91.60
16	86.89
17	90.97
18	84.75
19	94.32
20	92.10
21	93.93
22	92.66
23	90.62
24	84.06
25	94.57
26	87.00
27	87.84
28	90.92
29	92.49
30	91.27
31	91.99
32	86.44
33	85.30
34	94.97
35	83.45
36	94.46
37	91.42
38	88.96
39	94.13
40	83.91
41	88.77
42	92.41
43	88.68
44	88.82
45	93.05
46	84.14
47	94.29
48	83.02
49	84.52
50	92.99
51	90.04
52	83.77
53	94.84
54	94.86
55	87.76
56	90.73
57	86.10
58	92.56
59	85.63
60	91.04
61	87.20
62	87.15
63	93.57
64	92.39
65	92.31
66	89.54
67	85.18
68	86.12
69	86.50
70	83.35
71	91.67
72	84.51
73	85.70
74	93.70
75	94.19
76	91.72
77	87.49
78	92.75
79	86.77
80	88.44
81	83.91

**Table 2:** The actual measurement effect of the analysis model of factors affecting the export of film and television copyrights based on the gray correlation algorithm.

Number	Factor analysis
1	86.28
2	88.29
3	88.04
4	93.70
5	90.52
6	89.12
7	91.73
8	84.89
9	88.61
10	85.59
11	84.82
12	90.58
13	94.94
14	88.45
15	94.54
16	88.78
17	83.70
18	87.78
19	85.29
20	94.30
21	87.94
22	87.31
23	85.73
24	88.36
25	83.51
26	88.30
27	94.48
28	87.61
29	86.04
30	87.35
31	89.36
32	85.80
33	85.88
34	94.95
35	88.46
36	91.43
37	85.51
38	93.44
39	86.88
40	94.84
41	94.08
42	94.91
43	93.73
44	88.14
45	86.54
46	91.05
47	89.09
48	87.06
49	83.57
50	88.10
51	83.45
52	91.57
53	84.29
54	83.58
55	86.00
56	92.51
57	87.76
58	89.42
59	85.11
60	90.78
61	87.98
62	92.19
63	84.43
64	85.04
65	92.36
66	87.41
67	94.93
68	90.25
69	83.59
70	89.36
71	90.27
72	93.99
73	91.09
74	85.88
75	91.34
76	86.90
77	85.06
78	89.70
79	93.36
80	89.52
81	94.37

## Data Availability

The labeled dataset used to support the findings of this study is available from the corresponding author upon request.

## References

[1] Myers C. S. (2018). Plagiarism and copyright: b. *College & Undergraduate Libraries*.

[2] Rooksby J. H., Hayter C. S. (2019). Copyrights in higher education: motivating a research agenda. *The Journal of Technology Transfer*.

[3] Sharfina N. H., Paserangi H., Rasyid F. P., Fuady M. I. N. Copyright issues on the prank video on the youtube.

[4] Nekit K., Ulianova H., Kolodi D. (2019). Website as an object of legal protection by Ukrainian legislation. *Amazonia Investiga*.

[5] Lunyachek V., Ruban N. (2018). Managing intellectual property rights protection in the system of comprehensive seconday education. *Public Policy and Administration*.

[6] Schroff S. (2019). An alternative universe? Authors as copyright owners- the case of the Japanese Manga Industry. *Creative Industries Journal*.

[7] Finck M., Moscon V. (2019). Copyright law on b: between new forms of rights administration and digital rights management 2.0. *IIC - International Review of Intellectual Property and Competition Law*.

[8] Dharmawan N. K. S. (2017). Protecting traditional Balinese weaving trough copyright law: is it appropriate?. *Diponegoro Law Review*.

[9] McSherry J. P. (2018). The labor of literature: democracy and literary culture in modern Chile by jane D griffin. *Journal of Global South Studies*.

[10] Carugno G. (2018). How to protect traditional folk music? Some reflections upon traditional knowledge and copyright law. *International Journal for the Semiotics of Law - Revue internationale de Sémiotique juridique*.

[11] Matulionyte R. (2019). Empowering authors via fairer copyright contract law. *Law Journal*.

[12] Hudson E. (2017). The pastiche exception in copyright law: a case of mashed-up drafting?. *Intellectual Property Quarterly*.

[13] Sag M. (2019). The new legal landscape for text mining and machine learning. *Journal of the Copyright Society of the U.S.A*.

[14] Geiregat S. (2017). Digital exhaustion of copyright after CJEU judgment in Ranks and Vasiļevičs. *Computer Law & Security Report*.

[15] Slauter W. (2018). Introduction: copying and copyright, publishing practice and the law. *Victorian Periodicals Review*.

[16] Rosati E. (2017). The Monkey Selfie case and the concept of authorship: an EU perspective. *Journal of Intellectual Property Law & Practice*.

[17] Chatterjee I. (2021). Artificial intelligence and patentability: review and discussions. *International Journal of Modern Research*.

[18] Jongsma D. (2017). Parody after d - a comparative overview of the approach to parody under copyright law in Belgium, France, Germany and The Netherlands. *IIC - International Review of Intellectual Property and Competition Law*.

[19] Popescu I. G., Sechel G., Leaşu F. G. (2018). Biomedical research ethics. *Romanian Journal of Morphology and Embryology*.

[20] Rizzo S. G., Bertini F., Montesi D. (2019). Fine-grain watermarking for intellectual property protection. *EURASIP Journal on Information Security*.

[21] Vansover Y. (2019). On the natural aspect of historical thinking in the classroom. *International Journal of Innovation, Creativity and Change*.

